# Kinect-Based Rehabilitation Systems for Stroke Patients: A Scoping Review

**DOI:** 10.1155/2022/4339054

**Published:** 2022-03-27

**Authors:** Sohrab Almasi, Hossein Ahmadi, Farkhondeh Asadi, Leila Shahmoradi, Goli Arji, Mojtaba Alizadeh, Hoshang Kolivand

**Affiliations:** ^1^Department of Health Information Technology and Management, School of Allied Medical Sciences, Shahid Beheshti University of Medical Sciences, Tehran, Iran; ^2^Centre for Health Technology, University of Plymouth, Plymouth, UK; ^3^Health Information Management Department, School of Allied Medical Sciences, Tehran University of Medical Sciences, Tehran, Iran; ^4^Department of Health Information Technology, School of Nursing and Midwifery, Saveh University of Medical Sciences, Markaz, Iran; ^5^Department of Computer Engineering, Lorestan University, Khorramabad, Iran; ^6^School of Computer Science and Mathematics, Liverpool John Moores University, Liverpool, UK

## Abstract

**Method:**

This study was conducted according to Arksey and O'Malley's framework. To investigate the evidence on the effects of Kinect-based rehabilitation, a search was executed in five databases (Web of Science, PubMed, Cochrane Library, Scopus, and IEEE) from 2010 to 2020.

**Results:**

Thirty-three articles were finally selected by the inclusion criteria. Most of the studies had been conducted in the US (22%). In terms of the application of Kinect-based rehabilitation for stroke patients, most studies had focused on the rehabilitation of upper extremities (55%), followed by balance (27%). The majority of the studies had developed customized rehabilitation programs (36%) for the rehabilitation of stroke patients. Most of these studies had noted that the simultaneous use of Kinect-based rehabilitation and other physiotherapy methods has a more noticeable effect on performance improvement in patients.

**Conclusion:**

The simultaneous application of Kinect-based rehabilitation and other physiotherapy methods has a stronger effect on the performance improvement of stroke patients. Better effects can be achieved by designing Kinect-based rehabilitation programs tailored to the characteristics and abilities of stroke patients.

## 1. Introduction

Stroke is the second most prevalent cause of mortality and disability worldwide. The prevalence of stroke will increase due to the aging of the population. Moreover, stroke happens in a larger number of young populations in low- and middle-income communities [1]. It damages the sensory, motor, perception, visual, and cognitive systems, disrupts the patients' ability to conduct daily activities, and impacts their quality of life and level of independence [2, 3].

Rehabilitation in stroke is a purposeful process to help the patients regain and retain their social, intelligence, mental, and physical abilities while also helping them perform their daily and social activities with some level of independence [4, 5]. Rehabilitation exercises should include specific, repetitive, intensive, meaningful, and motivational tasks to improve the patients' motor performance [6]. Starting rehabilitation immediately after a stroke greatly contributes to patients' performance improvement, and effective rehabilitation depends on the patients' adherence to exercise programs and their regular performance at home and physiotherapy clinics. The process of rehabilitation in stroke patients is a long one, and patients' follow-up of this process is seriously limited due to its heavy costs, the long distance to rehabilitation centers, lack of access to such centers, patients' motor limitations, and problems associated with commuting to the health-care centers [6–8]. Moreover, patients' motivation for rehabilitation, which is a key factor for following the treatment and improving the outcome, is reduced because of the prolonged duration of rehabilitation [7].

The use of technology in rehabilitation is increasing rapidly. One of these technologies is video games, which is known as an effective intervention in rehabilitation. Video games are a useful solution for stroke patients who are unable to perform daily activities in the real environment and also motivate and encourage people to do rehabilitation exercises and improve motor function in stroke patients [8]. Video games are a new and useful technology that allows the user to interact with a three-dimensional environment. Studies have shown that this technology is an effective, safe, feasible solution that facilitates rehabilitation treatment [9]. In addition, video games increase motivation and increase patient satisfaction and involvement [10, 11]. Studies show that video games are used for a wide range of disorders including balance, cognition, mobility, and improved motor function. Video games are a promising tool because they provide the repetitive, task-based, reward-based, and interactive situations needed to restore patient function after brain injury [12]. Kinect-based video games are a good tool for providing rehabilitation exercises in the form of games due to the features of Kinect and the limitations of stroke patients [13, 14]. The application of Kinect-based rehabilitation as a low-cost and flexible method is rapidly expanding [15]. Kinect contains an RGB camera (R for red, G for green, and B for blue), a depth sensor, and a layer of microphones to record body movements and detect faces and voices [16]. Microsoft Kinect is a markless motion capture system that presents innovative and exciting methods for offering a more enjoyable treatment and promoting motivation in and adherence to the treatment [17, 18]. A unique feature of Kinect is providing a method for interaction with the game without using any controllable or wearable device [19, 20].

Another feature of Kinect for patients is performing rehabilitation exercises at home with no need for a physiotherapist [21]. By providing exciting and innovative rehabilitation methods, Kinect enhances adherence to treatment through adding entertaining features to the treatment, lessening costs compared to traditional rehabilitation, and making rehabilitation more accessible [17, 22]. Two types of games, commercial and customized, are used in Kinect-based rehabilitation. Some studies have utilized commercial Kinect-based games for rehabilitation. Although these games had positive effects on the performance improvement of stroke patients, since they had been developed for healthy people for entertainment purposes and required a high level of speed and ability, stroke patients could not easily perform them due to their limited and diverse abilities [8, 23]. On the other hand, some studies have developed games customized to the abilities of stroke patients. These games, known as serious games, were aimed for something beyond mere entertainment, and the results show that they positively affect the performance improvement of patients [24, 25].

Today, serious games, especially exergames, are used by therapists as a tool for rehabilitation purposes [26, 27]. Exergaming involves physical activity and is directly related to the sport in the game, not to the game or sport itself. Many studies have introduced exercise games in rehabilitation to motivate, engage, and increase patient adherence to their treatments [28, 29]. Research confirms the motivational benefits of using exergames in rehabilitation regardless of their age or illness [30].

Based on the findings of systematic reviews on the clinical and technical evaluation of the Kinect sensor, the use of this rehabilitation system is acceptable due to its cost-effectiveness and adequate precision in movement tracking [22, 31, 32]. Various studies have been conducted on the validity and accuracy of Kinect in tracking movements and the effect of Kinect on rehabilitation and motor recovery. Research on the validity and accuracy of the Kinect sensor indicates that this sensor has sufficient precision in movement tracking [20, 31, 33, 34]. Studies on the effects of Kinect on the performance improvement of patients with neurological disorders (such as Parkinson's disease and multiple sclerosis) have also deemed this method effective [17, 31, 32, 35].

The aim of scoping review is to determine, retrieve, and summarize the research pertinent to special issues to identify the key concepts supporting a research domain and the major sources and available evidence [36]. Scoping reviews are conducted to answer more general questions. One of their advantages is determining the feasibility and necessity of conducting a systematic review in a specific domain [36, 37]. So far, no comprehensive study has been conducted on Kinect-based rehabilitation for stroke patients. Therefore, this scoping review focused on the effects of Kinect-based rehabilitation for stroke patients and its limitations and challenges. Accordingly, the following research questions were posed:

1. What is the effect of Kinect-based rehabilitation systems on the performance of stroke patients?
2. What is the main application domain of a Kinect-based rehabilitation system for stroke patients?
3. What are the limitations of utilizing Kinect-based rehabilitation systems for stroke patients?

## 2. Methods

The current scoping review adopted Arksey and O'Malley's methodology [36]. Based on this framework, a scoping review has five essential steps and one selective step: (1) identification of the research question; (2) recognition of pertinent researches; (3) selection of studies; (4) charting the data; and 5) summarizing and disseminating the results and (6) consultation exercise. The sixth step was omitted in this review. This scoping review was conducted based on the Preferred Reporting Items for Systematic Reviews and Meta-Analyses Extension for Scoping Review (PRISMA-ScR) guidelines [38].

### 2.1. Eligibility Criteria

The main inclusion criteria for this review were as follows:

- English articles published in peer-reviewed journals and conferences with an available full text
- Articles published from 1 January 2010 to 13 October 2020
- Articles using Kinect-based rehabilitation for stroke patients
- Articles clinically evaluating and using Kinect for tracking movements and interactions in the rehabilitation system

### 2.2. Exclusion Criteria

Furthermore, the most important exclusion criteria for this review were as follows:

- Review articles, case reports, case studies or study protocols, letter to the editor, correspondences, and conference papers (absence or lack of access to the full text)
- Articles in languages other than English
- Articles merely evaluating the accuracy and validity of Kinect and not clinically evaluating the use of Kinect for improving the conditions of stroke patients
- Articles examining conditions other than stroke

### 2.3. Search Strategy and Information Sources

Articles were searched in five online databases (PubMed, Web of Science, Cochrane Library, IEEE Xplore, and Scopus). The search strategy comprised MeSH terms and other relevant keywords, and the two groups of terms were combined using Boolean operators AND and OR. The search was limited to the 2010-2020 period since Microsoft's first generation of Kinect sensors was introduced in November 2010 [10, 11]. The key terms used in this review was as follows: ((Stroke OR stroke rehabilitation) AND (Kinect OR Microsoft Kinect OR Xbox-Kinect OR virtual reality OR virtual reality exposure therapy OR virtual Reality exposure therapy OR virtual reality OR video games OR video games)). A summary of the characteristics of the included studies is provided in Table 1.

### 2.4. Study Selection

The electronic search was performed in the five mentioned databases. Also, hand-searching was performed in Google Scholar, and 58 articles were retrieved. The retrieved articles were then inputted to EndNote, and the duplicates were identified and removed by using the software. Subsequently, the titles and abstracts of the articles were reviewed by two authors according to the research questions and objectives. In the next step, the full text of the papers was examined by two authors concerning the inclusion and exclusion criteria. Any disagreements between the authors were resolved by discussions.

### 2.5. Data Extraction, Charting, and Synthesis

Data extraction was executed by using a form including the first author's name (reference), year of publication, country, the domain of rehabilitation, type of rehabilitation program (commercial vs. customized), main findings, and technical limitations of the Kinect-based rehabilitation program. The data were obtained by two authors, and disagreements were resolved upon discussions. Finally, the data extracted from the articles were inputted to Microsoft Excel for classification, synthesis, and reporting of the results.

## 3. Results

### 3.1. Selection of Sources of Evidence

Totally, 1196 articles were retrieved by searching in the databases. In the next step, by using EndNote, 184 duplicates were removed, and 954 articles remained. Subsequently, the titles and abstracts of the papers were reviewed, 856 papers were removed, and 98 remained. Then, the full text of the articles was examined, 64 articles were removed, and finally, 34 articles were included in this scoping review.  Figure 1 displays the article selection process.

### 3.2. Characteristics of the Sources of Evidence

The data extracted from the articles were recorded in the data extraction form (Table 1). The majority of the studies had been conducted in the US (*n* = 7, 22%), followed by Spain and South Korea (*n* = 5, 15%).

Following the invention of Kinect in 2010, the number of studies on the use of Kinect-based rehabilitation programs for stroke patients increased (Figure 2). However, no study based on the inclusion and exclusion criteria had been conducted in 2010, 2011, and 2014. The majority of the studies had been conducted in 2018 (*n* = 8).

### 3.3. Classification of the Studies Based on the Rehabilitation Domain

In the analysis of the domain of rehabilitation for stroke patients, most studies had focused on upper extremities (*n* = 22), followed by balance (*n* = 10), cognitive rehabilitation (*n* = 3), lower body (*n* = 2), and functional recovery (*n* = 2) (Figure 3).

In terms of the effects of Kinect-based rehabilitation programs, the majority of the studies had evaluated it as positive leading to the performance improvement of stroke patients [39–48]. Most studies had also mentioned that, compared to the use of routine treatment methods alone, the simultaneous application of Kinect-based rehabilitation and other physiotherapy methods has a stronger effect on the performance improvement of stroke patients [18, 24, 48–60].

Furthermore, the results revealed that the use of a Kinect-based rehabilitation program increases the repetitions of the movements, improves motivation, promotes the quality of life, and enhances adherence to treatment [18, 41–44, 46, 61, 62]. Some studies had employed telerehabilitation, reporting that Kinect-based rehabilitation is a safe and effective method for providing standard rehabilitation at home, whereby patients do not have to be present at physiotherapy clinics [59, 61, 63–66]. There was only one study in which the use of Kinect-based rehabilitation had the same effect on the intervention and control groups, and there was no difference between the two groups [67].

#### 3.3.1. Upper Extremities

The results of this study showed that 56% of the articles were in the field of upper limb rehabilitation. Patients' movements in the study were measured using Fugl-Meyer Assessment and Brunnstrom Motor Recovery Stage, which used Kinect-based rehabilitation games to improve patients' shoulder, elbow, wrist, and finger movements and ultimately to improve daily activities. There was an increase in patients' quality of life.

#### 3.3.2. Balance

The results of this study showed that 26% of the articles were in the field of balance rehabilitation. In the studies studied using Box and Block Test, Barthel Index, and Berg Balance Scale, it was measured that the use of Kinect-based rehabilitation games improved patients' balance.

#### 3.3.3. Cognitive Rehabilitation

The results of this study showed that 8% of the articles were in the field of cognitive rehabilitation. The results of the studies showed that the use of Kinect-based rehabilitation games improved patients' attention, spatial awareness, and generalized cognitive functioning.

#### 3.3.4. Lower Body

The results of this study showed that 5% of the articles were in the field of lower limb rehabilitation. In these studies, the Timed Up and Go Test and Fugl-Meyer Assessment erew used to measure lower limb movements, and the results showed that it improved lower limb movement.

### 3.4. Technical Limitations of Kinect-Based Rehabilitation Systems

In terms of the type of rehabilitation program used for stroke patients, the majority of the studies had designed the rehabilitation program tailored to the status and abilities of the patients (*n* = 13, 38%), while the other studies had utilized commercial Kinect-based programs (*n* = 21, 62%). Among the studies using commercial Kinect-based programs, technical limitations mostly included not challenging enough, lack of customization to the patients' abilities, complexity and difficulty of use, dependency on the therapist due to complexity, and the content of the programs being radically different from the daily activities of stroke patients [44, 48, 50, 53, 56, 68]. In the studies designing games customized to the abilities of stroke patients, technical limitations included the low speed of the games, the use of inappropriate feedback, insufficient precision of movement tracking, the complexity of games and difficulty of use, inappropriate user interface, dependence on the therapist, and not customized to and compatibility with the abilities of patients (Figure 4) [41, 47, 52, 54, 61, 65].

## 4. Discussion

This scoping review investigated the effect of using Kinect-based rehabilitation systems on the performance improvement of stroke patients, the rehabilitation domain, and technical limitations. The reviewed articles were published since 2010, when Microsoft-invented Kinect was examined [10, 11]. The results revealed that Kinect-based virtual rehabilitation leads to motor recovery in stroke patients. This type of rehabilitation is an effective and promising method owing to its low cost, flexibility, providing repetitive exercises, and motivation for the patients.

The most important feature of Kinect is that there is no need for any wearables during rehabilitation [20]. This feature of Kinect-based rehabilitation increases the repetitions of the movements, promotes motivation, enhances the quality of life, and increases adherence to treatment [18, 41–44, 46, 61, 62]. Moreover, due to its cost-effectiveness, flexibility, and telerehabilitation feature, the use of Kinect-based rehabilitation is a safe and effective method for providing standard rehabilitation at home [59, 61, 63–66]. The results of this study show that the use of Kinect-based rehabilitation games improves motor function in the upper and lower limbs and balance and improves cognitive function in improving stroke patients. These results are in line with the results of other similar studies in the field of using Kinect-based rehabilitation in improving the motor function of the upper [69], lower limbs [70], balance [71], and cognition [72].

Most studies had also mentioned that, compared to the use of routine treatment methods alone, the simultaneous application of Kinect-based rehabilitation and other physiotherapy methods has a stronger effect on the performance improvement of stroke patients. Regarding the positive outcome of simultaneous use of Kinect-based rehabilitation and other physiotherapy methods, the results of the present research are consistent with those of other papers [73, 74].

Despite all these advantages, some studies utilizing commercial Kinect-based programs reported different effects on the performance improvement of stroke patients; the reason was the limitations of these programs such as not challenging enough, not being customized to the patients' abilities, complexity, dependency on the therapist due to the complexity of the games, and the difference between the content of the games with patients' daily activities [43, 44, 50, 56, 57, 68]. Although some of these programs will be beneficial in combination with other rehabilitation methods, as they have been designed for the healthy population and entertainment purposes, they require rapid and difficult movements that may not be compatible with the abilities of stroke patients [23, 75].

On the other hand, some studies had developed games customized to the abilities of stroke patients and reported positive effects on their motor recovery [42, 50, 53, 56, 61, 62]. These results are in line with the findings of other researches [25, 73]. To promote the effects of Kinect-based rehabilitation programs, it is necessary to pay attention to the characteristics of the patients and their abilities in the program's development process. The use of clear feedback, presenting challenges appropriate for patients' abilities [60], telemonitoring patients by the therapist [20], using rewards [69], and including the socialization feature to induce a sense of competition between patients, is essential in this process.

To promote neural plasticity in rehabilitation programs, tailor-made rehabilitation systems are promising tools for patients. Furthermore, appropriate feedback should be provided to actively engage patients in better motor recovery. One of the essential elements in rehabilitation programs is to keep the patients motivated and engaged. In this way, caregivers should provide suitable feedback to correctly execute the exercise. The caregiver should change the different parameters of exercise to make it challenging and simultaneously possible for executing.

Since the therapist cannot regularly monitor and evaluate the patient's condition in Kinect-based rehabilitation systems, using different sensors such as brain and body wearable sensors can receive more data to help better assess the patient. Captured data should be interpreted and presented by utilizing graphs to simply be understood by physicians. To enhance the efficacy of rehabilitation systems, the user interface should be designed by considering both patients' restrictions and caregivers' needs.

## 5. Limitations and Future Directions

One limitation of the current study was the diversity in the type of studies and the small samples of some studies, which pose problems in drawing definitive conclusions about the positive effects of Kinect-based rehabilitation on the motor recovery of stroke patients. Lack of access to the full text of some papers was another limitation. About the positive effect of customized Kinect-based rehabilitation programs which are tailored to the abilities of stroke patients, it is suggested more research be conducted on the design framework of such programs and their effects on the motor recovery of stroke patients. Furthermore, developing the rehabilitation systems should concentrate on a range of complex factors such as patients living environment, social environment, different challenges of daily living, and patients' skills in using various technologies. Furthermore, developing systems with a concentration on supporting personal goals and performing the rehabilitative exercise in a competitive atmosphere may increase progress over time. It will be necessary to conduct different clinical trials in large sample size, as well as different devices to determine which factors have a greater effect in achieving a better outcome. Furthermore, performing a meta-analysis study to investigate whether rehabilitation programs are beneficial in improving patients function in stroke is essential.

## 6. Conclusion

Because of some limitations such as the costs of rehabilitation, the long distance to rehabilitation centers, lack of access to such centers, patients' motor limitations, and commute problems, patients with stroke lose motivation to follow treatment. The application of Kinect-based rehabilitation is an effective solution for creating motivation and improving adherence to rehabilitation programs in stroke patients. Kinect-based rehabilitation will be more effective on the performance improvement of these patients if used as a complementary technique in combination with other rehabilitation methods. Furthermore, to promote effects on motor recovery, it is essential to pay attention to the design of rehabilitation programs customized to the abilities of stroke patients.

## Figures and Tables

**Figure 1:** Scoping review flowchart.

**Figure 2:** Distribution of the research papers based on publication year.

**Figure 3:** Distribution of the papers based on rehabilitation domain.

**Figure 4:** Distribution of the papers based on technical limitations.

**Table 1:** A summary of the characteristics of the included studies.

#	First author (Ref)	Year	Country	Rehabilitation domain	Type of rehabilitation program	Number of sessions	Duration (week)	Outcome measures (mean (SD))	Key findings	Technical limitations
1	Sheehy [68]	2020	Canada	Balance and UE rehabilitation	Commercial game	10-12	4	Experimental group: pre/post differences for FIST were 3.4 (confidence interval [CI] 0.5; 6.3) Control group: pre/post differences for FIST were 5.3 (2.9; 7.7)	The improvement in balance and upper extremities was the same in the intervention and control groups, and there was no difference between the two groups.	The Kinect-based rehabilitation program not being challenging and customized to the users' abilities
2	Shahmoradi [67]	2020	Iran	UE rehabilitation	Customized game	10	4	Games have positive effects on the horizontal abduction of shoulder (16.26 ± 23.94, *P* = 0.02), horizontal adduction of shoulder (59.24 ± 74.76, *P* = 0.01), supination of wrist (10.68 ± 53.52, *P* = 0.02), elbow flexion (0.1 ± 1.5, *P* = 0.01), and wrist flexion (0.06 ± 1.34, *P* = 0.03).	Kinect-based rehabilitation improved the upper extremity range of motion.	No game being designed for fingers due to an imprecise Kinect sensor and no patient progress reporting feature in the software
3	Norouzi-Gheidari [49]	2020	Canada	UE rehabilitation	Customized game	10	4	The efficacy measures showed statistically meaningful improvements in the activities of daily living measures (i.e., MAL-QOM (motor activity log-quality of movement) and both mobility and physical domains of the SIS (stroke impact scale) with mean difference of 1.0%, 5.5%, and 6.7% between the intervention and control group, respectively) at postintervention.	Compared to the use of routine treatment methods alone, the simultaneous application of Kinect-based rehabilitation and other physiotherapy methods has a stronger effect on the performance improvement of upper extremities.	Not mentioned
4	Maier [39]	2020	Spain	Cognitive rehabilitation	Customized game	10	6	The experimental group showed improvements in attention (*P* < .01), spatial awareness (*P* < .01), and generalized cognitive functioning (*P* < .001).	Kinect-based rehabilitation has positive effects on stroke patients' attention, spatial awareness, and depression.	Not mentioned
5	Cano-Mañas [50]	2020	Spain	Balance rehabilitation	Commercial game	40	5	Modified Rankin scores (*P* < 0.01) and the Barthel index (*P* < 0.01).	The combination of Kinect-based rehabilitation and other physiotherapy methods improves patients' balance, performance, and motivation.	Commercial Kinect-based games are not designed specifically for stroke patients, and it is difficult to adapt them to the patients' abilities
6	Mokhtar [40]	2019	Egypt	UE rehabilitation	Customized game	18	6	The modified Barthel index score for the study group (*P* < 0.05). Grip muscle strength for the study group (*P* < 0.05). The modified Barthel index score for the control group at the end of the treatment was significantly lower than in the study group (*P* < 0.05).	Kinect-based rehabilitation improves upper extremity performance.	Not mentioned
7	Ho [51]	2019	Taiwan	Functional recovery	Customized game	7	1	Functional outcomes (mRS improvement from the baseline; − 0.58 vs. − 0.23, *P* < 0.001) and reduced medical cost (Taiwan dollar; 49474 vs. 66306, *P* < 0.005).	Compared to the use of routine treatment methods alone, the simultaneous application of Kinect-based rehabilitation and other physiotherapy methods has a stronger effect on the performance improvement of stroke patients.	Not mentioned
8	Foreman [41]	2019	USA	UE rehabilitation	Customized game	1	—	High dose of reaching repetitions (461 ± 184), with an average of 81% being successful and 19% involving compensatory trunk flexion.	Kinect-based rehabilitation program increases the repetitions of movements, enhances motivation, and leads to upper extremity performance improvement in stroke patients.	(1) The games are slow and there is no patient progress reporting feature (2) Displaying the feedbacks is not appropriate for some patients. Providing sound feedbacks, using a larger monitor, and keeping the appropriate distance from the Kinect sensor are better for patients with visual impairment (3) Tracking with Kinect sensor is not completely reliable. It does not precisely track some movements, causes problems in interaction with games, and leads to incorrect feedback
9	Boone [42]	2019	USA	UE rehabilitation	Customized game	24	12	Fugl-Meyer Assessment; preintervention (34.4 ± 10.6); postintervention (42.7 ± 10.4).	Kinect-based rehabilitation program increases the repetitions of movements, enhances motivation, and leads to upper extremity performance improvement in stroke patients.	Not mentioned
10	Aramaki [43]	2019	Brazil	Functional recovery	Commercial game	36	12	COPM; pretest performance: 2.12 (0.81). COPM; posttest performance: 6.40 (1.82) (*P* < 0.001) COPM; pretest satisfaction: 1.64 (0.88) COPM; posttest satisfaction: 6.22 (1.78) (*P* < 0.001)	Kinect-based rehabilitation program is an appropriate tool for patients' performance improvement, increasing their motivation, and enhancing their treatment adherence.	Not mentioned
11	Adomavičienė [76]	2019	Lithuania	UE and cognitive rehabilitation	Customized game	10	2	Self-care (*P* < 0.05). Decreased muscle tone, improved shoulder and elbow ROMs, hand dexterity, and grip strength (*P* < 0.05). Anxiety level (*P* < 0.05).	Kinect-based rehabilitation improves the upper extremity performance and cognitive ability.	Not mentioned
12	Triandafilou [61]	2018	USA	UE rehabilitation	Customized game	9	3	Arm displacement averaged 350 m for each VERGE training session.	Kinect-based rehabilitation increases the movements and patients' motivation and is an effective tool for rehabilitation at home.	The complex scenario of the games requires high cognitive abilities and causes problems in patients' learning and coordination
13	Schaham [44]	2018	Israel	UE and LE rehabilitation	Commercial game	4-22	12	—	Kinect-based rehabilitation is an appropriate tool for rehabilitation, increases patients' motivation, and leads to performance improvement.	Commercial Kinect-based games that are not designed specifically for stroke patients sometimes cause problems for patients in controlling and learning the games
14	Liao [45]	2018	USA	UE rehabilitation	Customized game	15	5	Fugl-Meyer Assessment scores (*P* = 0.001). Wolf Motor Function Test (*P* = 0.008). Active range of motion (*P* < 0.05). Stroke impact scale-hand function (*P* = 0.016).	Kinect-based rehabilitation improves the upper extremity performance of stroke patients.	Not mentioned
15	Kim [52]	2018	South Korea	UE rehabilitation	Customized game	50	10	FMA: sham (46.8 ± 16.0) and the real VR group (49.4 ± 14.2) (*P* = .937 in intention to treat analysis).	Kinect-based rehabilitation will be more effective if used in combination with other physiotherapy methods.	(1) The activities in the games are not similar to the patients' real-life tasks (2) Due to the games' poor user interface, the patients depend on the physiotherapist for selecting the type of game compatible with their abilities
16	Ikbali Afsar [53]	2018	Turkey	UE rehabilitation	Commercial game	20	4	At posttreatment, a statistically significant increase was found in both groups in the upper extremity and hand Brunnstrom stages, FMAUE, FIM self-care subscore, and BBT score (*P* < .001).	Kinect-based rehabilitation will be more effective if used in combination with other physiotherapy methods.	Commercial Kinect-based games are not designed specifically for stroke patients, and it is difficult to adapt the games to the patients' abilities
17	Held [63]	2018	Switzerland	Balance rehabilitation	Customized game	36	12	—	Kinect-based rehabilitation is a safe and effective method of providing standard rehabilitation at home.	Not mentioned
18	Grigoras [54]	2018	Romania	UE rehabilitation	Customized game	12	3	FMA (*P* = 0.039).	Kinect-based rehabilitation will be more effective if used in combination with other physiotherapy methods.	The game cannot be played at home in the absence of a physiotherapist and without training due to its advanced features
19	Aşkın [55]	2018	Turkey	UE rehabilitation	Customized game	20	5	FMA (*P* < 0.05). BBT (*P* < 0.05). Motricity index (*P* < 0.05).	Kinect-based rehabilitation will be more effective if used in combination with other physiotherapy methods.	Not mentioned
20	Türkbey [56]	2017	Turkey	UE rehabilitation	Commercial game	20	5	BBT (*P* < 0.005). WMFT—performance time score (*P* < 0.005). WMFT—functional ability score (*P* < 0.005). FIM self-care score (*P* < 0.018). BMRS—upper extremity (*P* < 0.010).	Kinect-based rehabilitation is a safe and reliable method for upper extremity performance improvement and will be more effective if used in combination with other physiotherapy methods.	Commercial Kinect-based games are not designed specifically for stroke patients, and it is difficult to adapt the games to the patients' abilities
21	Park [57]	2017	South Korea	LE and balance rehabilitation	Commercial game	42	6	FMS (*P* < 0.005). BBT (*P* < 0.005). TUG (*P* < 0.005).	Kinect-based rehabilitation will be more effective if used in combination with other physiotherapy methods.	Commercial Kinect-based games are not designed specifically for stroke patients, and it is difficult to adapt the games to the patients' abilities
22	Moldovan [46]	2017	Romania	UE and balance rehabilitation	Customized game	10	2	Final ARAT score improved from 46 to 57 points (24% amendment), the Fugl-Meyer test score improved from 46 to 52 (13% amendment), and the Berg Balance Scale improved from 43 to 49 points (14% amendment).	Kinect-based rehabilitation improves patients' upper extremity performance, balance, and treatment adherence.	Not mentioned
23	Maier [47]	2017	Spain	Cognitive rehabilitation	Customized game	10	2	—	Kinect-based rehabilitation is a novel and promising approach to cognitive rehabilitation.	Kinect-based rehabilitation programs could not be adapted to the patients' cognitive abilities
24	Lee [48]	2017	Taiwan	Balance rehabilitation	Commercial game	12	6	BS (*P* = 0.001). TUG-cog test (*P* = 0.005).	Kinect-based rehabilitation is an effective method for balance improvement and will be more effective if used in combination with other physiotherapy methods.	Commercial Kinect-based games are not designed specifically for stroke patients, and it is difficult to adapt the games to the patients' abilities.
25	Tsoupikova [62]	2016	USA	UE rehabilitation	Customized game	9	3	—	Kinect-based rehabilitation improves patients' upper extremity performance and adherence to treatment.	Not mentioned
26	Lai [64]	2016	Taiwan	Balance rehabilitation	Customized game	10	2	BBS (*P* < 0.005).	Kinect-based rehabilitation improves patients' balance and adherence to treatment and can be used at home.	Not mentioned
27	Shin [58]	2015	South Korea	UE rehabilitation	Customized game	20	5	FMA (*P* < 0.079). Emotional problems (*P* = 0.047). Depression (*P* = 0.017). Upper extremity function (*P* = 0.001)	If used in combination with other physiotherapy methods, Kinect-based rehabilitation will lead to upper extremity performance improvement in stroke patients.	Not mentioned
28	Proffitt [65]	2015	USA	UE rehabilitation	Customized game	30	6	FMA (*P* < 0.05)	Kinect-based rehabilitation is a cost-effective, safe, and effective method for performance improvement of stroke patients and can be used at home.	(1) No choice to the type of game (2) Not displaying more feedbacks on the monitor (3) Lack of a *help* feature for troubleshooting and solving technical issues (4) Poor user interface and problems with findings the icons
29	Lloréns [18]	2015	Spain	Balance rehabilitation	Customized game	36	12	Berg Balance Scale (*ηp*(2) = .68; *P* = .001). Balance (*ηp*(2) = .24; *P* = .006). Gait (*ηp*(2) = .57; *P* = .001).	The combination of Kinect-based rehabilitation and other physiotherapy methods improves patients' balance and adherence to treatment.	Not mentioned
30	Brokaw [24]	2015	USA	UE rehabilitation	Customized game	20	4	Stroke Impact Scale-16; before: 67 after: 68. Fugl-Meyer; before: 34 after:39. Shoulder; before: 17 after: 19. Wrist; before: 6 after: 6. Hand; before: 11 after: 14.	The combination of Kinect-based rehabilitation and other physiotherapy methods improves patients' upper extremity performance and adherence to treatment.	Not mentioned
31	Singh [66]	2014	Malaysia	Balance rehabilitation	Commercial game	12	6	Timed Up and Go Test; F (1, 26) = 5.83, *P* = 0.02; and the 30-second Sit to Stand test; F (1, 26) = 13.50, *P* = 0.001.	As a complementary technique in combination with other physiotherapy methods, Kinect-based rehabilitation leads to performance improvement and can be used at home.	Not mentioned
32	Sin [59]	2013	South Korea	UE rehabilitation	Commercial game	12	6	FMA (*P* < 0.05). BBS (*P* < 0.05).	The combination of Kinect-based rehabilitation and other physiotherapy methods improves patients' upper extremity performance and adherence to treatment.	Not mentioned
33	Lee [8]	2013	South Korea	UE rehabilitation	Commercial game	18	6	FMA (*P* < 0.05)	The combination of Kinect-based rehabilitation and other physiotherapy methods improves patients' upper extremity performance and adherence to treatment.	Not mentioned
34	Wiederhold [60]	2012	Spain	Balance rehabilitation	Commercial game	20	4	BBS (*P* < 0.05)	Kinect-based rehabilitation is an effective tool that improves the balance of stroke patients.	Not mentioned

UE: upper extremity; LE: lower extremity; COPM: Canadian Occupational Performance Measure; BBT: Box and Block Test; FIM: Functional Independence Measure; FMA: Fugl-Meyer Assessment; WMFT: Wolf Motor Function Test; BMRS: Brunnstrom Motor Recovery Stage; TUG: Timed Up and Go Test; ARAT: Action Research Arm Test; BBS: Berg Balance Scale.

## Additional Points

*Key messages.* (i) Kinect-based rehabilitation is an effective and promising solution that improves the motivation, adherence to treatment, and motor function of stroke patients. (ii) Compared to the use of routine treatment methods alone, the simultaneous application of Kinect-based rehabilitation and other physiotherapy methods has a stronger effect on the performance improvement of stroke patients. (iii) Kinect-based rehabilitation programs developed based on the abilities of stroke patients have more pronounced effects on performance improvement compared to commercial Kinect-based programs.
